# Novel Value of Preoperative Gamma-Glutamyltransferase Levels in the Prognosis of AFP-Negative Hepatocellular Carcinoma

**DOI:** 10.1155/2020/4269460

**Published:** 2020-07-10

**Authors:** Liang-He Lu, Wei-Wei, Anna Kan, Jie-Mei, Yi-Hong Ling, Shao-Hua Li, Rong-Ping Guo

**Affiliations:** ^1^Department of Hepatobiliary Oncology, Sun Yat-sen University Cancer Center, China; ^2^State Key Laboratory of Oncology in South China, China; ^3^Collaborative Innovation Center for Cancer Medicine, Guangzhou 510060, China; ^4^Department of Pathology, Sun Yat-sen University Cancer Center, China

## Abstract

**Background:**

Gamma-glutamyltransferase (GGT) is involved in tumor development and progression, but its prognostic value in *α*-fetoprotein- (AFP-) negative (AFP < 25 ng/mL) hepatocellular carcinoma (HCC) patients remains unknown.

**Methods:**

A large cohort of 678 patients with AFP-negative HCC following curative resection who had complete data were enrolled in this study. The optimal cutoff value for the preoperative level of GGT was determined by the X-tile program. Independent prognostic factors for overall survival (OS) and disease-free survival (DFS) were also identified.

**Results:**

The optimal cutoff values for the preoperative levels of GGT were 37.2 U/L and 102.8 U/L, which were used to divide all patients into three subgroups (group 1, GGT < 37.2 U/L (*n* = 211, 31.1%); group 2, GGT ≥ 37.2 and <102.8 U/L (*n* = 320, 47.2%); group 3, GGT ≥ 102.8 U/L (*n* = 147, 21.7%)), with distinct OS times (58.5 vs. 53.5 vs. 44.4 months, *P* < 0.001) and DFS times (47.9 vs. 40.3 vs. 30.1 months, *P* < 0.001). Elevated preoperative GGT levels were associated with an unfavorable tumor burden (larger tumor size, multiple tumors, and microvascular invasion) and were selected as independent predictors of a worse OS (group 2 vs. group 1, HR: 1.73 (1.13-2.65), *P* = 0.011; group 3 vs. group 1, HR: 3.28 (2.10-5.13), *P* < 0.001) and DFS (group 2 vs. group 1, HR: 1.52 (1.13-2.05), *P* = 0.006; group 3 vs. group 1, HR: 2.11 (1.49-2.98), *P* < 0.001) in multivariable analysis.

**Conclusions:**

Elevated preoperative GGT levels are associated with an unfavorable tumor burden and serve as an independent prognostic marker for worse outcomes in AFP-negative HCC patients following resection.

## 1. Introduction

Hepatocellular carcinoma (HCC) is one of the most common and aggressive human malignancies in the world and the third leading cause of cancer-related death worldwide [1]. The prognosis of HCC patients remains unsatisfactory due to the extremely high incidence of recurrence after curative resection [2, 3]. Currently, the universal blood biomarker used for the risk assessment and surveillance of HCC is serum *α*-fetoprotein (AFP), but nearly 30% of HCC patients have a normal serum level of AFP (AFP < 25 ng/mL) [4–7]. Data regarding the characteristics and outcomes of patients with tumors that do not produce AFP are limited. Finding another reliable biomarker and identifying factors that allow better stratification of AFP-negative patients with worse outcomes would be beneficial in clinical practice.

Gamma-glutamyltransferase (GGT) is found predominantly on the surface of secretory epithelial cells [8]. Abnormal GGT expression has been reported to play a role in tumor progression, invasion, and anticancer drug resistance [9, 10] and is associated with worse prognosis in several human tumors, including ovarian cancer [11], cervical cancer [12], and endometrial cancer [13]. Large epidemiological studies revealed that high serum levels of GGT are associated with an increased risk of liver cancer [14, 15]. Elevated GGT levels have been reported to be a predictor of poor prognosis in HCC patients [16–19]. However, further analysis of the utility of preoperative levels of GGT in AFP-negative HCC patients is lacking.

Therefore, the specific aim of our study was to evaluate the prognostic value of preoperative GGT in AFP-negative HCC patients after resection.

## 2. Materials and Methods

This study protocol was conducted in accordance with the ethical guidelines of the 1975 Declaration of Helsinki, and the procedure was approved by the institutional review board of the Sun Yat-sen University Cancer Center. Informed consent was obtained from each patient included in the study. The study was censored on 31 December 2017.

### 2.1. Study Population

The inclusion criteria for patients in this study were as follows: (1) patients with histologic confirmation of HCC; (2) age between 18 and 75 years; (3) AFP < 25 ng/mL; (4) albumin-bilirubin (ALBI) grade [20, 21] 1 or 2; (5) Eastern Cooperative Oncology Group performance status 0; and (6) resectable disease defined as the complete removal of all macroscopic tumor tissue and retention of a liver remnant sufficient to sustain life, as assessed by our surgical team [22]. The exclusion criteria were as follows: (1) palliative tumor resection, (2) incomplete clinical data, (3) loss to follow-up within three months after resection, and (4) patients with a history of previous anticancer therapy before resection. In total, we enrolled 678 consecutive HCC patients who underwent primary curative resection from December 2004 to December 2013 at Sun Yat-sen University Cancer Center.

### 2.2. Preoperative Measurement of the Serum Level of GGT

The normal limit for GGT in our center ranges from 10 to 60 U/L. In all cases, data including demographics and clinical, biological, radiological, and treatment outcomes were prospectively collected. The measurement of the level of GGT was performed within 3 days prior to surgery, and the maximum values were used when multiple values were available.

### 2.3. Hepatic Resection

Hepatic resection was carried out as we have described previously [6, 23]. To assess the number and size of the lesions and the relationship of the tumors to vascular structures, intraoperative ultrasonography was performed routinely. Pringle's maneuver was used to occlude the blood inflow of the liver. A clamp-crushing method was utilized for liver resection. Our preferred surgical method for multiple nodules in one segment or in neighboring segments was anatomic resection with en bloc resection. For multiple bilobar nodules, anatomic resection was preferred for the main tumor, whereas satellite nodules were resected nonanatomically with a negative resection margin. Nonanatomic resection with a negative resection margin was performed if an inadequate liver remnant would have been created. A negative resection margin was defined as the lack of visible tumor cells in the margins of the remnant liver closest to the gross edge of the tumor.

### 2.4. Follow-Up

Follow-up examinations consisted of physical examinations, serum AFP tests, liver function tests, and at least one imaging examination, including abdominal ultrasonography, contrast-enhanced computed tomography (CT), or magnetic resonance imaging (MRI). Most patients were scheduled for follow-up visits once every 3 months for the first two years and then every 3 to 6 months thereafter. Recurrence was defined as the appearance of a new lesion with the radiological features of HCC after resection. For patients in whom tumor recurrence was detected, the choice of treatment was based on the EASL-EORTC clinical practice guidelines and determined by a multidisciplinary team [24].

### 2.5. Statistical Analysis

The optimal cutoff point for the preoperative serum level of GGT was determined by the X-tile program [25]. The main end point of the study was overall survival (OS), which was defined as the interval from the date of resection until death or the end of the follow-up period. The second end point was disease-free survival (DFS), which was defined as the interval from the date of resection until the first recurrence or the last follow-up visit. Categorical variables were compared using the chi-square test or Fisher's exact test, and one-way ANOVA was performed for continuous variables. Survival curves were estimated using the Kaplan-Meier method and analyzed with log-rank tests. Cox proportional hazard models were used to identify factors associated with the OS and DFS. The regression coefficients (*B*) of the Cox regression model were multiplied by 2 and rounded to the nearest unit (1.00 units) to obtain simple point numbers to facilitate the bedside calculation of the GGT-based prognostic score (GBPS). Statistical analyses were performed using IBM SPSS v.19.0 (SPSS, Armonk, NY, USA). A two-tailed *P* value less than 0.05 was considered statistically significant.

## 3. Results

### 3.1. Patient Characteristics

As the cutoff points for preoperative GGT varied greatly in previous studies, ranging from 17.9 to 165 U/mL and to avoid an arbitrary cutoff point, all patients were divided into the following three subgroups using X-tile v.3.6.1 software (Yale University, New Haven, CT): group 1 was composed of patients with preoperative levels of GGT < 37.2 U/L (*n* = 211, 31.1%), group 2 was composed of patients with preoperative levels of GGT ≥ 37.2 and <102.8 U/L (*n* = 320, 47.2%), and group 3 was composed of patients with preoperative levels of GGT ≥ 102.8 U/L (*n* = 147, 21.7%) (Figures 1(a) and 1(b)). The clinicopathologic characteristics are summarized in Table 1. Elevated preoperative serum GGT levels were associated with unfavorable tumor burden, including larger tumor size, multiple tumor number, and microvascular invasion (MVI) (Table 1). A total of 609 (89.8%) patients were classified as BCLC grade A, while 45 (6.6%) patients were classified as grade B, and 24 (3.6%) patients were classified as grade C. At the time of censoring, 219 patients (32.3%) had died of HCC, including 32 patients (15.2%) in group 1, 86 patients (26.9%) in group 2, and 67 patients (45.6%) in group 3. During the follow-up period, HCC recurrence was identified in 68 patients (32.2%) in group 1, 161 patients (50.3%) in group 2, and 83 patients (56.5%) in group 3.

### 3.2. Significant Factors Affecting Overall Survival

The 1-, 3-, and 5-year OS rates were 97.2%, 75.4%, and 44.5% in group 1; 92.5%, 69.1%, and 39.7% in group 2; and 89.1%, 55.8%, and 27.2% in group 3, respectively (Figure 1(c)) (all *P* < 0.001). Univariate analysis of OS is shown in Table 2, and parameters with *P* < 0.05, including alanine aminotransferase (ALT) level, total bilirubin level (TBIL), albumin level, GGT level, ALBI grade, liver cirrhosis, tumor size, tumor number, and MVI, were included in multivariate analysis using Cox proportional hazards regression analysis. Only the TBIL level, GGT level, ALBI grade, tumor number, and MVI remained significant predictors of OS (Figure 2).

### 3.3. Significant Factors Affecting Disease-Free Survival

The 1-, 3-, and 5-year DFS rates were 88.2%, 59.2%, and 33.6% in group 1; 74.7%, 49.4%, and 24.7% in group 2; and 66.6%, 34.0%, and 15.6% in group 3, respectively (Figure 1(d)) (all *P* < 0.001). In univariate analysis of DFS, significant differences were observed in the following variables: HBV/HCV, ALT level, GGT level, ALBI grade, tumor size, tumor number, and MVI (Table 2). The results of the multivariate analysis using the Cox proportional hazards regression analysis are shown in Figure 3. HBV/HCV, GGT level, tumor size, tumor number, and MVI remained significant independent prognostic indicators for DFS.

### 3.4. Subgroup Analysis according to Milan Criteria and Microvascular Invasion

As an increased preoperative GGT level was associated with unfavorable tumor burden, we further evaluated OS and DFS by stratifying patients according to the Milan criteria and MVI (Figure 4). Among the subgroups of patients within or beyond the bounds of the Milan criteria, preoperative GGT levels divided all patients into three groups with significantly different OS (both *P* < 0.001) (Figures 4(a) and 4(c)) and DFS (*P* < 0.001, *P* = 0.023, respectively) (Figures 4(b) and 4(d)). When the subgroup of patients with MVI was stratified according to preoperative GGT level, significant differences in OS were not found (*P* = 0.299) (Figure 4(e)), while the DFS of patients in group 2 and group 3 overlapped (*P* = 0.037) (Figure 4(f)); however, when the subgroup of patients without MVI was stratified according to preoperative GGT levels, the OS and DFS were significantly different (both *P* < 0.001) (Figures 4(g) and 4(h)). For patients with BCLC grade A, preoperative GGT levels can be used to stratify all patients into three groups with significantly different OS and DFS (both *P* < 0.001) (Figures 4(i) and 4(j)).

### 3.5. A New Scoring System Based on GGT Level

To predict the prognosis of AFP-negative HCC patients, parameters recognized as significant in the multivariate analysis were used to form the GGT-based prognostic score (GBPS) as follows: GBPS = TBIL (≤17.2 = 0; >17.2 = 1) + GGT (≤37.2 = 0; 37.2‐102.8 = 1; ≥102.8 = 2) + ALBI (grade 1 = 0; grade 2 = 1) + cirrhosis (absent = 0; present = 1) + tumor number (≤1 = 0; >1 = 2) + MVI (absent = 0; present = 2). We used the X-tile program and showed that the optimal cutoff points of the GBPS score were 2 and 5. The entire cohort was then divided into three subgroups (≤2; 2-5; >5), which had significantly different OS (5-year OS rate: 89.4%, 69.6%, 35.6%, respectively; *P* < 0.001) and DFS (5-year DFS rate: 67.2%, 47.4%, 21.7%, respectively; *P* < 0.001) (Figures 5(a) and 5(b)). The GBPS model had a higher area under the curve value than the TNM stage and BCLC stage for AFP-negative HCC patients (0.726, 0.664, 0.569) (Figure 5(c)).

## 4. Discussion

Although serum AFP is a well-established prognostic marker in HCC, nearly one-third of HCC patients are AFP-negative. Our study showed that preoperative GGT levels can be employed as another effective marker to replace AFP as a predictor of prognosis in AFP-negative HCC patients, helping stratify the AFP-negative HCC patients who are at high risk of death and early recurrence. Moreover, the measurement of GGT is reliable and inexpensive and extensively applied in clinical practice.

Hu et al. reported that high serum levels of GGT are associated with an increased risk of liver cancer [14]. Zhang et al. and Guiu et al. found that the GGT level served as an important prognostic factor in patients with intermediate HCC treated with TACE [17, 19]. Ma et al. reported that the serum level of GGT was a convenient prognostic marker for OS and recurrence in HCC patients undergoing RFA [18]. Fu et al. reported that GGT was a promising and reliable prognostic marker in patients following liver transplantation [16]. The cutoff values of preoperative GGT in patients with HCC varied in these studies. Although molecular markers predicting HCC prognosis have been studied extensively [5, 26–28], data on the outcomes in AFP-negative HCC patients are limited.

Using the cutoff points of 37.2 U/L and 102.8 U/L determined with the X-tile program, we divided AFP-negative HCC patients into three groups with distant prognoses. In this study, we demonstrated that the preoperative level of GGT is associated with unfavorable tumor factors, including larger tumor size, multiple tumor number, and MVI, which was consistent with the findings of previous studies on gynecological cancer. Tumor size and tumor number are both independent risk factors for HCC. The prognosis of patients worsened when tumor size and tumor number increased. Defining tumor characteristics that exceed the Milan criteria that significantly impact the prognosis of HCC after resection is thus important. Additionally, previous studies showed that the presence of MVI indicated aggressive behavior of HCC and predicted a worse prognosis after liver resection [29, 30]. The early spread of cancer cells via the vasculature may be a key mechanism underlying metastasis and recurrence. However, some patients without MVI still suffer tumor recurrence shortly after curative resection in clinical practice. Thus, considering the imbalance of the baseline characteristics and to avoid being overly assertive, we further evaluated the prognostic role of the preoperative level of GGT in the subgroup of patients who met the Milan criteria and had MVI. The results showed that the preoperative GGT level was able to accurately stratify patients according to their risk level in both the subgroups of patients meeting and exceeding the Milan criteria. For patients without MVI, the preoperative GGT level may serve as a complementary marker for prognostic stratification.

As a principal enzyme involved in glutathione metabolism, GGT can exert prooxidative effects at the membrane surface and in the extracellular microenvironment. Preceding studies described GGT as contributing to persistent oxidative stress, which is a factor in genomic instability [31] and modulation of the process involved in tumor progression [9, 32]. Another theory is that GGT is induced by inflammatory cytokines, such as tumor necrosis factor-*α* and interferon [33], which are involved in carcinogenetic processes and the regulation of the tumor microenvironment [34, 35]. However, the mechanisms underlying the association between preoperative GGT and the prognosis of patients with HCC remain unclear and require further basic research.

Because this was a retrospective study, certain biases might exist. We enrolled a large cohort of 678 patients to address this limitation. Second, as the majority of patients had evidence of HBV infection, our data require validation in other study groups in whom HCV infection is the prevailing etiology of chronic liver disease.

In conclusion, the preoperative GGT level serves as a feasible prognostic factor for AFP-negative HCC patients following resection.

## Figures and Tables

**Figure 1:** The cutoff points of the preoperative GGT level in AFP-negative HCC patients using X-tile plots. Group 1 was defined as GGT < 37.2 U/L; group 2: GGT ≥ 37.2 and <102.8 U/L; group 3: GGT ≥ 102.8 U/L. (a) The cutoff points are highlighted by black/white circles. (b) The three subgroups are indicated on a histogram including the entire cohort. (c) A Kaplan-Meier curve of overall survival (group 1 vs. group 2 vs. group 3, 58.5 vs. 53.5 vs. 44.4 months, all *P* < 0.001). (d) A Kaplan-Meier curve of disease-free survival (group 1 vs. group 2 vs. group 3, 47.9 vs. 40.3 vs. 30.1 months, all *P* < 0.001).

**Figure 2:** Multivariate analysis and forest plot of the hazard ratio of risk factors for overall survival. OS: overall survival; HR: hazard ratio; CI: confidence interval; TBIL: total bilirubin; GGT: gamma-glutamyltransferase; ALBI grade: albumin-bilirubin grade; MVI: microvascular invasion.

**Figure 3:** Multivariate analysis and forest plot of the hazard ratio of risk factors for disease-free survival. DFS: disease-free survival; HR: hazard ratio; CI: confidence interval; HBV: hepatitis B virus; HCV: hepatitis C virus; GGT: gamma-glutamyltransferase; MVI: microvascular invasion.

**Figure 4:** Subgroup analyses based on the Milan criteria and MVI. Group 1 was defined as GGT < 37.2 U/L; group 2: GGT ≥ 37.2 and <102.8 U/L; group 3: GGT ≥ 102.8 U/L. The overall survival (a) and disease-free survival (b) curves of patients meeting the Milan criteria. The overall survival (c) and disease-free survival (d) curves of patients exceeding the Milan criteria. The overall survival (e) and disease-free (f) curves of patients with microvascular invasion. The overall survival (g) and disease-free survival (h) curves of patients without microvascular invasion. The overall survival (i) and the disease-free survival (j) curves of patients classified as BCLC grade A.

**Figure 5:** GGT-based prognostic score (GBPS). (a) Overall survival and (b) disease-free survival curves. (c) AUC values for GBPS, TNM stage, and BCLC stage.

**Table 1:** Clinical characteristics of patients.

Variables	GGT < 37.2 U/L (*n* = 211)	GGT ≤ 37.2 U/L and GGT < 102.8 U/L (*n* = 320)	GGT ≥ 102.8 U/L (*n* = 147)	*P* value
Age (years)	52.0 ± 12.3	53.4 ± 10.8	50.7 ± 11.2	0.060
Sex				<0.001
Male	181 (85.8)	305 (95.3)	142 (96.6)	
Female	30 (14.2)	15 (4.7)	5 (3.4)	
Cause of disease				0.702
HBV	179 (84.8)	278 (86.9)	126 (85.7)	
HCV	2 (0.9)	7 (2.2)	4 (2.7)	
Others	31 (14.7)	40 (12.5)	19 (12.9)	
Platelet count (10^9^/L)	173.9 ± 58.5	175.4 ± 68.1	183.1 ± 89.5	0.448
Liver cirrhosis				0.167
Present	112 (53.1)	195 (60.9)	89 (60.5)	
Absent	99 (46.9)	125 (39.1)	58 (39.5)	
Albumin (g/L)	42.5 ± 3.3	41.9 ± 4.0	41.5 ± 4.2	0.051
Serum total bilirubin (*μ*mol/L)	13.9 ± 5.6	14.2 ± 5.8	14.8 ± 8.5	0.424
ALBI grade				
1	183 (86.7)	254 (79.4)	115 (78.2)	0.055
2	28 (13.3)	66 (20.6)	32 (21.8)	
Tumor size (cm)	4.3 ± 2.3	5.4 ± 2.7	6.7 ± 3.5	<0.001
Tumor number				0.009
≤1	190 (90.0)	263 (82.2)	116 (78.9)	
>1	21 (10.0)	57 (17.8)	31 (21.1)	
Tumor extent				0.119
Unilobar	206 (97.6)	303 (94.7)	137 (93.2)	
Bilobar	5 (2.4)	17 (5.3)	10 (6.8)	
Microvascular invasion				0.001
Absent	189 (89.6)	268 (83.8)	109 (74.1)	
Present	22 (10.4)	52 (16.2)	38 (25.9)	
Surgical time (min)	165.6 ± 60.6	169.5 ± 52.9	179.5 ± 55.6	0.065
Type of hepatectomy^†^				0.107
Major	36 (17.1)	61 (19.1)	38 (25.9)	
Minor	175 (82.9)	259 (80.9)	109 (74.1)	
Surgical margin^‡^ (cm)				0.062
<1	73 (34.6)	136 (42.5)	68 (46.3)	
≥1	138 (65.4)	184 (57.5)	79 (53.7)	
Intraoperative blood loss (mL)				<0.001
<400	160 (75.8)	217 (67.8)	71 (48.3)	
≥400	51 (24.2)	103 (32.2)	76 (51.7)	
Encapsulation				0.414
Complete	104 (49.3)	149 (46.6)	62 (42.2)	
Incomplete	107 (50.7)	171 (53.4)	85 (57.8)	
Tumor differentiation				0.235
Well	48 (22.7)	57 (17.8)	24 (16.3)	
Moderate or poor	163 (77.3)	263 (82.2)	123 (83.7)	
BCLC stage				<0.001
A	200 (94.8)	288 (90.0)	121 (82.3)	
B	10 (4.7)	27 (8.4)	8 (5.4)	
C	1 (0.5)	5 (1.6)	18 (12.3)	

Variables are expressed as no. (%). HBV: hepatitis B virus; HCV: hepatitis C virus; ALBI grade: albumin-bilirubin grade; BCLC: Barcelona Clinic Liver Cancer. ^†^Major liver resection: resection with more than two lobes; minor liver resection: resection with no more than two lobes. ^‡^Surgical margin: the shortest measured distance from the edge of the tumor to the plane of liver transection.

**Table 2:** Univariate analysis of risk factors for overall survival and disease-free survival.

Variables	OS		DFS	
	HR (95% CI)	*P*	HR (95% CI)	*P*
Age (y)				
≤50	Reference		Reference	
>50	1.19 (0.88-1.61)	0.251	1.09 (0.87-1.37)	0.458
Gender				
Female	Reference		Reference	
Male	1.03 (0.60-1.78)	0.905	0.83 (0.53-1.30)	0.415
Etiology				
Other	Reference		Reference	
HBV/HCV	1.37 (0.85-2.21)	0.192	1.91 (1.28-2.85)	0.002
PLT (10^9^/L)				
>100	Reference		Reference	
≤100	1.35 (0.88-2.05)	0.166	1.28 (0.92-1.79)	0.149
ALT (U/L)				
≤40	Reference		Reference	
>40	1.37 (1.03-1.83)	0.032	1.47 (1.18-1.84)	0.001
TBIL (*μ*mol/L)				
≤17.2	Reference		Reference	
>17.2	1.39 (1.00-1.90)	0.044	1.19 (0.93-1.53)	0.174
Albumin (g/L)				
>35	Reference		Reference	
≤35	3.45 (1.70-7.02)	0.001	0.84 (0.31-2.24)	0.720
GGT (U/L)				
≤37.2	Reference		Reference	
37.2-102.8	1.94 (1.29-2.91)	0.001	1.82 (1.37-2.42)	<0.001
≥102.8	3.92 (2.57-5.99)	<0.001	2.53 (1.84-3.49)	<0.001
ALBI grade				
1	Reference		Reference	
2	1.92 (1.39-2.67)	<0.001	1.32 (1.00-1.75)	0.048
Liver cirrhosis				
No	Reference		Reference	
Yes	1.41 (1.04-1.92)	0.027	1.22 (0.97-1.54)	0.086
Tumor size, cm				
≤5	Reference		Reference	
>5	1.84 (1.37-2.47)	<0.001	1.61 (1.28-2.00)	<0.001
Tumor number				
≤1	Reference		Reference	
>1	3.20 (2.35-4.36)	<0.001	2.01 (1.59-2.72)	<0.001
MVI				
Absent	Reference		Reference	
Present	2.61 (1.86-3.67)	<0.001	1.96 (1.48-2.59)	<0.001

OS: overall survival; DFS: disease-free survival; PLT: platelet; ALT: alanine aminotransferase; TBIL: total bilirubin; GGT: gamma-glutamyltransferase; ALBI grade: albumin-bilirubin grade; MVI: microvascular invasion.

## Data Availability

Key raw data in our study have been uploaded onto the Research Data Deposit public platform (http://www.researchdata.org.cn/) with the approval number as RDDA2019001105.

## Abbreviations

HCC: Hepatocellular carcinoma
AFP: *α*-Fetoprotein
GGT: Gamma-glutamyltransferase
TACE: Transcatheter arterial chemoembolization
RFA: Radiofrequency ablation
LT: Liver transplantation
ALBI grade: Albumin-bilirubin grade
CT: Contrast-enhanced computed tomography
MRI: Magnetic resonance imaging
OS: Overall survival
DFS: Disease-free survival
MVI: Microvascular invasion
ALT: Alanine aminotransferase
TBIL: Total bilirubin.
